The article "Pneumonia Detection Using an Improved Algorithm Based on Faster R-CNN" was published in 2021. Journal: Comput Math Methods Med.

# Pneumonia Detection Using an Improved Algorithm Based on Faster R-CNN

**DOI:** 10.1155/2021/8854892

**Published:** 2021-04-21

**Authors:** Shangjie Yao, Yaowu Chen, Xiang Tian, Rongxin Jiang

**Affiliations:** ^1^Institute of Advanced Digital Technology and Instrumentation, Zhejiang University, Zhejiang 310027, China; ^2^Zhejiang Provincial Key Laboratory for Network Multimedia Technologies, Zhejiang University, Zhejiang 310027, China; ^3^Institute of Advanced Digital Technology and Instrumentation, Zhejiang University and State Key Laboratory of Industrial Control Technology, Zhejiang University, Zhejiang 310027, China

## Abstract

Pneumonia remains a threat to human health; the coronavirus disease 2019 (COVID-19) that began at the end of 2019 had a major impact on the world. It is still raging in many countries and has caused great losses to people's lives and property. In this paper, we present a method based on DeepConv-DilatedNet of identifying and localizing pneumonia in chest X-ray (CXR) images. Two-stage detector Faster R-CNN is adopted as the structure of a network. Feature Pyramid Network (FPN) is integrated into the residual neural network of a dilated bottleneck so that the deep features are expanded to preserve the deep feature and position information of the object. In the case of DeepConv-DilatedNet, the deconvolution network is used to restore high-level feature maps into its original size, and the target information is further retained. On the other hand, DeepConv-DilatedNet uses a popular fully convolution architecture with computation shared on the entire image. Then, Soft-NMS is used to screen boxes and ensure sample quality. Also, K-Means++ is used to generate anchor boxes to improve the localization accuracy. The algorithm obtained 39.23% Mean Average Precision (mAP) on the X-ray image dataset from the Radiological Society of North America (RSNA) and got 38.02% Mean Average Precision (mAP) on the ChestX-ray14 dataset, surpassing other detection algorithms. So, in this paper, an improved algorithm that can provide doctors with location information of pneumonia lesions is proposed.

## 1. Introduction

According to a study by Liu et al. [1] in 2015, among the 5.9 million deaths of children under 5, over 15.6% were due to pneumonia; timely diagnosis and treatment could greatly reduce this mortality level. However, the contrast in chest X-ray [2] images is low, making manual evaluation inefficient [3]. Computer-aided diagnosis [4] can enhance efficiency and lead to timely treatment.

The size, shape, and position of pneumonia can vary a great deal [5]. Its target contour is very vague, which leads to great difficulty with detection, and enhancing the accuracy of detection is a major research problem. At present, detection algorithms include two-stage object detectors such as Faster R-CNN and one-stage detectors such as YOLO and SSD. The latter uses an additional stage to complete the task of multiscale target detection. They are faster than two-stage detectors but less accurate. Medical testing has high requirements for accuracy, and two-stage detectors have an advantage in this respect.

The article "Pneumonia Detection Using an Improved Algorithm Based on Faster R-CNN" was published in 2021. Journal: Comput Math Methods Med.

However, there are still problems with the backbone network of the current detection algorithms. For example, VGG and ResNet generally have two problems: a large network depth leading to long training time and massive downsampling that leads to the target position and semantic information being lost [6]. The goal is to assess using a deep feature map, since such a map has a large receptive field and the corresponding anchor is also large. However, the deeper the map, the lower the object-edge resolution, which reduces the assessment accuracy of the regression curve. In the low-resolution feature map, after continuous downsampling, the semantic features of the small target disappear in the deep layer; the semantic information of the large target is also partially lost, and the position will move, which is not conducive to accurate target detection. Usually, the way to optimize a network, such as GoogLeNet [7], is to extend its depth or width, but this generates huge numbers of parameters, easily leads to overfitting, and requires large amounts of tagged data to train.

Traditional deep networks reduce partial information when extracting features, and this affects their capacities for detection. The residual neural network structure of the low-complexity dilated bottleneck adopted in this paper avoids the computational lag associated with network depth and the problems involved in the large numbers of parameters associated with network width and integrates into the FPN [8] network. Extracting deep feature semantic information from an image, thereby avoiding loss of information, the Soft-NMS [9] operation is performed on props generated by the RPN; useful information is retained while filtering the extra box, and finally, a model able to detect pneumonia to a high level of precision is obtained.

## 2. Related Studies

### 2.1. Object Detection Works

In 2016, Redmon et al. [10] proposed YOLO, which does not require a separate region proposal network, so its detection speed is extremely fast and can reach 45 FPS. In the same year, Liu et al. [11] proposed the SSD algorithm. Both SSD and YOLO win in detection speed, but SSD uses a multiscale feature map to detect independently, the spatial resolution of images in deep networks has been significantly reduced, and it may not be possible to locate small targets that are difficult to detect in low resolution, reducing the accuracy of detection. YOLO does not use multiscale feature maps for independent detection. It smoothes the feature map and splices it with another lower-resolution feature map, but it treats the detection only as a regression problem and the detection accuracy is low. In 2014, Girshick et al. proposed R-CNN, which greatly improved the speed of training. On the PASCAL VOC 2010 dataset, the mAP improved from 35.1% to 53.7%. In 2015, Ren [12] and others proposed the Faster R-CNN algorithm, which uses RPN (region proposal network) to generate proposals on the feature map.

The article "Pneumonia Detection Using an Improved Algorithm Based on Faster R-CNN" was published in 2021. Journal: Comput Math Methods Med.

In 2018, Lee et al. [13] proposed DetNet, which was designed specifically for target detection and achieved better detection results with fewer layers. To avoid the large computational complexity and memory consumption caused by the high-resolution feature map, the network adopts a low-complexity dilated bottleneck structure; a higher resolution of the feature map is ensured while obtaining a higher subtractive field. This paper draws on the idea of DetNet and the framework of Faster R-CNN to study the detection of pneumonia.

### 2.2. Pneumonia Detection Works

In recent years, many scholars have made efforts to detect pneumonia. Abiyev and Ma'aitah [14] apply a convolutional neural network (CNN) for the diagnosis of chest X-ray diseases. Compared to BPNN and RNN, CNN gets higher precision but longer training time. Vijendran and Dubey [15] combine multilayer extreme learning machine (MLELM) and online sequential extreme learning machines (OSELM) to detect pneumonia on the chest X-ray image. Abiyev and Ma'aitah [14] explore the features extracted from layers of the CNN along with a set of classical features, including GIST and bag of words on a dataset of more than 600 radiographs.

The above algorithms performed well in the detection of pneumonia, but the amount and size of data involved are not large, and then, some scholars used a large amount of data on the deep network to do research. Jaiswal et al. [16] predicted potential pneumonia on the RSNA (Radiological Society of North America) dataset by Mask R-CNN, and the intersection over union-based mAP achieves 21.8%. Guendel et al. [17] proposed to use the DenseNet to solve the detective on the chest X-ray dataset. Chakraborty et al. [18] design a convolutional neural network architecture which contains a 17-layer network and many dense layers. It achieves 95.62% AP on the dataset of chest X-ray. Wang et al. [19] add unified weakly supervised multilabel image classification and disease localization framework in a deep convolutional neural network to solve the problems in ChestX-ray8. These mentioned approaches have been adjusted on the structure of the network, but not for improvements on the backbone. A backbone that is specifically for detection only is needed.

The article "Pneumonia Detection Using an Improved Algorithm Based on Faster R-CNN" was published in 2021. Journal: Comput Math Methods Med.

The COVID-19 pneumonia epidemic that broke out at the end of 2019 still threatens the survival of all mankind. At the same time, because of the rapid rate of infection of new crown pneumonia, how to quickly detect new crown pneumonia has placed great demands on the global medical system. Deep learning assists in the diagnosis of new crowns. Pneumonia research has proposed many methods. In 2020, Wang and Wong [20] proposed COVID-Net, which is a deep convolutional neural network design tailored for the detection of COVID-19 cases from chest X-ray (CXR) images. Mangal et al. [21] proposed CovidAID: COVID-19 AI Detector, which is a novel deep neural network-based model to triage patients for appropriate testing. Ozturk et al. [22] proposed a new model for automatic COVID-19 detection using raw chest X-ray images; this model is used to provide accurate diagnostics for binary classification (COVID vs. no findings) and multiclass classification (COVID vs. no findings vs. pneumonia). The accuracy of the former is 98.08%, and that of the latter is 87.02%. However, these studies only performed classification tasks and finally obtained an assessment of the probability of disease on the X-ray, and there was no way to detect the location information of the lesion.

## 3. Methodology

In this part, we introduce in detail our proposed DeepConv-DilatedNet method, including the data processing, the architecture of our network, and the effective enhancement effect of Soft-NMS.

### 3.1. Data Processing

In 2018, the Radiological Society of North America (RSNA) [b20] released a dataset on the detection and localization of pneumonia in chest X-rays [71]. The dataset is from the National Institutes of Health (National Institutes of Health) [48] public chest X-ray images, with radiologist [72] annotations. The detailed information of the RSNA pneumonia detection dataset can be found on the Kaggle website [73]. The RSNA pneumonia data used in this experiment contains data of 26684 cases, of which only 6012 pneumonia images (accounting for 22.03%), and the remaining 8851 normal images (accounting for 31.19%) and 11821 images (accounting for 44.77%), an image that is abnormal or has no turbidity in the lungs. In most deep learning, images without targets are of no use to the training of the network, so this part of the meaningless data is eliminated in the initial stage. Since the patient's chest pneumonia may have more than one location, there may be one to four locations. Therefore, in order to maintain sample balance, we finally use 6012 images with annotations, of which 4/5 is selected as the training set and 1/5 as the test set. And count the number of lesions in the training set and test set as shown in Table 1.

The article "Pneumonia Detection Using an Improved Algorithm Based on Faster R-CNN" was published in 2021. Journal: Comput Math Methods Med.

The images in training sets are augmented by flipping horizontally and vertically as shown in Figure 1. Finally, 14428 training images are acquired.

This paper analyzes the pixel characteristics of the pneumonia site. Pneumonia is considered to be slightly more opaque than its surroundings. All 6012 images have pneumonia; among them, 3265 cases have two areas of pneumonia, which accounted for the largest proportion in the dataset. There is an area in 2617 images, three areas in 118 cases, and four areas in 12 cases. Pneumonia is usually distributed in the left and right lobes, and its grayscale is blurred, which is difficult to identify directly [23]. The histogram of the average gray value distribution of the target area is shown in Figure 2. The image is first subjected to gradation, and then, the target area is cut. A gradation mean value statistic is performed on the target area being cut, and the average gradation value of each target area is obtained by reading the gradation value of each pixel and then averaging. The analysis shows that the gray values are concentrated between 50 and 200, a very wide range, making manual observation time-consuming and labor-intensive. Therefore, it is important to put to use the end-to-end method of deep learning.

Due to the characteristics of low brightness and low contrast of the chest X-ray image, to better detect the target area of pneumonia and improve the detection accuracy, the chest X-ray image can be preprocessed. In X-ray images, normal lungs will not absorb X-rays, so it will appear black. The location of the pneumonia is a gray dashed shadow or a cloudy area. To improve the recognition rate, contrast and brightness enhancement operations can be performed on X-ray images. In this article, the CLAHE algorithm is used to equalize the gray histogram to enhance contrast and brightness. The images before and after processing are shown in Figure 3.

To improve the effect of model training, it is necessary to enhance the training set. At first, we used the CLAHE algorithm to equalize the gray histogram of 6012 pictures with pneumonia given by RSNA, to enhance contrast and brightness. And then, the target area of pneumonia in every picture is used as a positive sample, and the remaining areas are used as a negative sample for training. Among them, 80% of samples, about 4810 pictures, are used as the training set, and 1202 pictures are used as the test set. The training set has less data, so it is increased by data enhancement. After horizontal flipping and vertical flipping, we finally get 14430 pictures as the training set.

The article "Pneumonia Detection Using an Improved Algorithm Based on Faster R-CNN" was published in 2021. Journal: Comput Math Methods Med.

### 3.2. Function of Convolution

The calculation equation of the convolutional neural network is shown in

(1) $$\begin{array}{c} N=\frac{\left(W-F+2P\right)}{S}+1, \end{array}$$

where *N* is the output size, *W* is the input size, *F* is the convolution kernel size, *P* is the padding value, and *S* is the stride value. For example, we input an RGB image, the size of our input image is 227 × 227 × 3, that is, it has three channels, and the size of each channel is 277∗277. We set the padding as 0 and the stride as 4, and then, the convolution kernel size is 3∗3. Through Formula (1), we can calculate the output size as *N* = (227 − 3 + 2 × 0)/4 + 1 = 57. Generally speaking, the larger the convolution kernel, the larger the receptive field, the more image information you can see, and the better the features you can obtain. That being said, a large convolution kernel will cause a surge in calculations, which is not conducive to the increase of model depth, and calculation performance will also decrease. Therefore, better features can be obtained by mixing convolution kernels of different sizes. In this paper, 1∗1, 3∗3, and 7∗7 convolution kernels were used to get better feature maps.

### 3.3. Detecting Pneumonia Using Deep Learning

The size of the anchor box will directly affect the detection performance of the model. This article analyzes the target area of the training data of the pneumonia X-ray dataset. In the traditional Faster R-CNN algorithm, the size of the anchor box depends on empiricism. Therefore, this article refers to the method of generating the anchor box in YOLOV3 and uses the K-Means++ algorithm to determine the aspect ratio suitable for the dataset. In this study, the K-Means++ algorithm is used to analyze the target region of the training set, and the pneumonia anchor box with three scales of [72, 73], [102, 120], and [140, 279] were generated. So the scale ratio of the anchor box was set to 0.5, 1.0, and 1.5.

FPN combines low-level and high-level features to obtain feature sets that can reflect multidimensional information. Researchers use upsampling to recover the original size feature map from high-level feature maps. Upsampling is an algorithm that restores an image to its original size. But deconvolution is another way to resize feature maps.  Figure 4 demonstrates that deconvolution can keep more features than upsampling.

All the current state-of-the-art image classification networks are convolutional networks, such as ResNet and GoogLeNet. Of note, the target detection network can be implemented using a fully convolutional network. Therefore, we design the DeepConv-DilatedNet that the fully connected layer and upsample layers are replaced by convolution layers.

The article "Pneumonia Detection Using an Improved Algorithm Based on Faster R-CNN" was published in 2021. Journal: Comput Math Methods Med.

The deep-learning pneumonia-detection method used in this paper is based on the Faster R-CNN, in which the backbone uses the low-complexity dilated bottleneck residual neural network called DeepConv-DilatedNet.

In the DetNet network, the first four phases of the backbone are consistent with the original ResNet50 phase, maintaining a 16x receptive field from the fifth stage and adding a stage, using 1 × 1 convolutions and 3 × 3 dilated convolutions in the fifth and sixth stages. The mapping performs channel superposition to form a bottleneck structure that expands the receptive field. Starting from the fourth stage, a different bottleneck structure is used to increase the receptive field and keep the feature layer dimension 256 unchanged, thus reducing the number of weight parameters. Adaptive average pooling is used throughout the network.

To enhance the pictorial information output of the DetNet network, this paper combines FPN and DetNet to enhance the feature-extraction mode of the network. And put forward the DeepConv-DilatedNet. DeepConv-DilatedNet removes the fully connected layer and only uses the convolutional layers to compute feature maps, speeding up the network. Meanwhile, we remove the upsample layers in FPN, and deconvolution is used to upsample the feature maps in FPN. The DeepConv-DilatedNet is shown in Figure 5.

The RPN generates a large number of anchor boxes through the sliding window, with many overlapping parts between them. In this paper, the Soft-NMS literature is used to filter the overlapping anchor boxes, as in Formula (2). For example, *i* ⊂ *M* is the label of the box, and the IoU value corresponding to *bi*, as an input to the function, is finally multiplied by *S*_*i*_ as the score of *bi* in the final box. After the screening is completed, RoI align pooling is performed; the feature map after the pooling process is input to the fully connected layer, and finally, the detection box and category of the target are output.

(2) $$\begin{array}{c} S_{i}=S_{i}e^{-}\frac{\text{IoU}{\left(M,bi\right)}^{2}}{\sigma }. \end{array}$$

### 3.4. Soft-NMS

In the process of target detection, whether using a sliding window or an RPN, many duplicate candidate frames will be generated. Therefore, even in the most advanced detectors, nonmaximum suppression algorithms are used to obtain the final detection set because it greatly reduces the number of false alarms. The core idea is an iterative-traversal-elimination process, and the low-scoring frame with an overlap rate greater than a fixed threshold will be suppressed by the high-scoring frame.

The article "Pneumonia Detection Using an Improved Algorithm Based on Faster R-CNN" was published in 2021. Journal: Comput Math Methods Med.

However, the traditional NMS method uses hard decisions to determine which candidate frames are retained or suppressed. Therefore, an object appears in the overlapping area of another object. That is, when two target frames are close, the frame with a lower score will be ignored. The overlapping area is too large and is deleted, which causes the detection of the object to fail and reduces the average detection rate of the algorithm. In this case, the detection algorithm should have output two detection frames, but the traditional nonmaximum value suppression algorithm will be filtered out because the score of one frame is low and the IoU of the two frames is greater than the set threshold. A target was detected. Therefore, it is necessary to use Soft-NMS, instead of simply and rudely setting the NMS to zero the score of the box whose IoU with the highest score is greater than the threshold, but replacing the original score with a slightly smaller score. Experiments also show that in a single model, Soft-NMS can increase the target detection result from 39.8% to 40.9% [9].

### 3.5. Our Method

For target detection, first, we chose the two-stage model Faster R-CNN with a suitable detection effect as the prediction framework, and then, we considered the excellent effect of DetNet59 as the backbone, so we used DetNet59 for the feature extraction of the target. But because DetNet59 upsampling will lose features, we improve DetNet59 and change upsampling to deconvolution to reduce feature loss, and at the same time, add hole convolution to expand the receptive field. Besides, the initial anchor box has a great influence on the training and prediction of the model, so we borrowed from the YOLO method and used the K-Means++ algorithm to obtain the initial anchor box for the pneumonia target dataset to improve the detection effect. Finally, because Soft-NMS improves the performance of the target detection network, we have joined Soft-NMS. Finally, we get the DeepConv-DilatedNet+Faster R-CNN shown as Figure 6.

## 4. Experiments

### 4.1. Training

In the beginning, we did not filter the initial RSNA dataset, so the dataset is full of many useless images, and the prediction effect of the model trained using such a dataset is very poor. After screening the dataset, the dataset without data enhancement is used to train the model, but because the amount of data was too small, the model could not fully converge and the prediction effect was not good. Finally, we reprocessed the dataset and got the current model training results.

The article "Pneumonia Detection Using an Improved Algorithm Based on Faster R-CNN" was published in 2021. Journal: Comput Math Methods Med.

The experiments were performed on the NVIDIA GeForce GTX 1080 configuration. With Cuda acceleration, processing 2 images per batch, the initial learning rate is set to 0.001, and the 10th epoch is reduced tenfold using the SGD optimization algorithm. The RPN bounding box regression uses the Smooth L1 loss function, and the classification uses the binary cross-entropy (CE) loss function.

To verify the effectiveness of the proposed method, we trained and evaluated four different backbones. The number of iterations exceeded 90000, and the model appeared to be stable. We plotted the classification and regression with the total loss curve for each model presented in Figure 7. The loss value of DeepConv-DilatedNet converges stably in the range of 0.4 to 0.5. The fitting effect is ideal. The loss value of DetNet59 and ResNet50 becomes gradually stable at around 0.24. The smooth drop of VGG16 is finally stabilized at 0.25; the fluctuation of ResNet101 becomes marginally stable at around 0.45, with a poor-fitting effect.

### 4.2. Evaluation Metrics

The IoU-threshold-based Average Precision (AP) value is utilized to illustrate the detection results. IoU is the overlap rate between the prediction box and the ground truth box. As seen in Formula (3), AP refers to the average score of each picture.

(3) $$\begin{array}{c} \text{AP}\left(S,i\right)=\frac{\Sigma_{i}S_{i}}{N}, \end{array}$$

(4) $$\begin{array}{c} \text{IoU}\left(\text{Pred},\text{GT}\right)=\frac{\text{Pred}⋂\text{ GT}}{\text{Pred}⋃\text{ GT}}. \end{array}$$

In Formula (4), Pred is the prediction box, GT refers to the ground truth box, where *S* presents the score of each testing picture and *N* specifies the number of all test pictures. Suppose IoU threshold is equal to a certain threshold when the predicted image's IoU threshold is more than or equal to the threshold; otherwise, *S* is 0.

(5) $$\begin{array}{c} \text{mAP}\left(p,t\right)=\frac{\Sigma_{t}p_{t}}{n}. \end{array}$$

In this paper, the Mean Average Precision (mAP) is used to describe the whole model's detection accuracy, such as in Formula (5), *t* refers to the threshold of IoU and the AP value at threshold *t* is *p*. *n* refers to the number of classes, so in this paper *n* = 1.

(6) $$\begin{array}{c} \text{FPR}=\frac{\text{FP}}{\text{FP}+\text{TN}}, \end{array}$$

(7) $$\begin{array}{c} \text{TPR}=\frac{\text{TP}}{\text{TP}+\text{FN}}. \end{array}$$

ROC is a tool for measuring nonequilibrium in classification [24], and its abscissa is the false-positive rate (FPR) as shown in Formula (6), and the ordinate is a true-positive rate (TPR) as shown in Formula (7). ROC curves are often used to evaluate the pros and cons of a binary classifier. The closer the ROC curve is to the upper left corner, the higher the true-positive rate obtained by the classifier in comparison to its false-positive rate, indicating that the classifier performs well.

The article "Pneumonia Detection Using an Improved Algorithm Based on Faster R-CNN" was published in 2021. Journal: Comput Math Methods Med.

To more fully verify the experimental results, we calculated the AUC (area under the curve) value [25]. AUC is a probability value. When positive and negative examples are randomly selected, the probability that the current classification algorithm ranks the positive instances ahead of the negative based on the calculated score is the AUC value. Therefore, the larger the AUC value, the more likely the classification algorithm is to rank positive examples ahead of negative ones, which makes for better classification.

### 4.3. Experimental Result

In experiments, a comparison of four different backbone AP indexes with different IoU thresholds is made, and the mAP values (*t* ∈ 0.4,0.5,0.6,0.7) are calculated as shown in Table 2. Firstly, comparing the detection effect of the model using DetNet59 as the backbone and the method using Vgg16, ResNet50, and ResNet101 as the backbone, respectively, we found that the effect of using DetNet59 as the backbone model is significantly better than others. Then, we compare our improved network with DetNet59; the result shows that our method is better than DetNet59. As can be seen from Table 2, the Faster R-CNN with DeepConv-DilatedNet as the backbone is higher than the DetNet59, ResNet50, ResNet 101, and VGG16 network models on each AP with different thresholds. On the RSNA dataset, DeepConv-DilatedNet reached 0.4570 at AP@0.5.

Next, we use Soft-NMS to filter the anchor box in the DeepConv-DilatedNet-based Faster R-CNN, with the model optimized for greater detection accuracy, as shown in Table 3. The same optimization of the other four networks leads to a detection performance that is still lower than that of DeepConv-DilatedNet, and DeepConv-DilatedNet has a clear advantage in terms of accuracy of detection of the IoU threshold of 0.4 to 0.5, which is 2.0175% more than the DetNet59 in the mAP index, 4.6325% more than ResNet50, and 5.465% more than VGG16. The results show that Soft-NMS can effectively improve the performance of target detection.

Besides, we plotted the specific changes of the AP value of the network in IoU ∈ [0, 1], as shown in Figure 8. The optimization effect of Soft-NMS is very obvious when IoU ∈ [0.5,0.6].

Furthermore, we compared our work with that of others, as shown in Table 4. MS is the mean score for every image overall threshold (ranges from 0.4 to 0.75 at a step size of 0.05) values; our result is 10.9% higher than those obtained by Abiyev and Ma'aitah [14] using Mask R-CNN, which shows that our model is reliable for detecting pneumonia.

The article "Pneumonia Detection Using an Improved Algorithm Based on Faster R-CNN" was published in 2021. Journal: Comput Math Methods Med.

To further verify the validity of the model, we also plot the ROC curve, as shown in Figure 9. The AUCs of DeepConv-DilatedNet and DetNet59 are 0.81 and 0.74, respectively; the AUC value of DeepConv-DilatedNet is 10% higher than that of DetNet59. A low false-positive rate yields higher sensitivity, which indicates that, compared with the traditional DetNet network, the subtle complexity dilated bottleneck is a very efficient feature extractor for detection tasks.

The PR line (precision/recall curve) of the five models shown in Figure 10 shows that the DeepConv-DilatedNet has excellent accuracy and recall rates.

We compare the detection effects of all methods on different quantities of ROI areas, as shown in Figure 11. No matter single target or multiple targets, the detection effects of our model are preferable to those of other benchmark models. The detection box is closer to the real target, and the number of detection boxes on the target box is closer and more accurate.

To know the usefulness of our model, we test our method on the ChestX-ray14 dataset. The ChestX-ray14 dataset contains 30805 patients and 112,120 chest X-ray images. The size of each image is 1024 × 1024 with 8 bits grayscale values. The corresponding report includes 14 pathology classes. There are 120 pneumonia images with bounding box annotations in ChestX-ray14. We choose all of them to check our model. From the result shown in Table 5, we can see the detection effect of DeepConv-DilatedNet is still better than other models.

## 5. Conclusion

In this paper, a low complexity residual neural network with a dilated bottleneck structure, called DeepConv-DilatedNet, is invoked as the backbone of a two-stage detector using Faster R-CNN. Because of the turbidity of the pneumonia target, the image has further been enhanced with the CLAHE algorithm to make the target area more prominent. In the RPN, we use the Soft-NMS algorithm to filter the anchor box and ensure its quality. To speed up the convergence of the algorithm and improve the prediction accuracy of the target area, we also used the K-Means++ algorithm in YOLOV3 to obtain the initial anchor box size. We implant deconvolutions in FPN to variance in scale and thus facilitate recognition from features computed on a single input scale. Finally, we got the result of this method. Combining the different sets of work done in each network, the ability of the algorithm to detect pneumonia accurately in the RSNA dataset is enhanced. To verify the validity of the model, we also compared it in detail with the traditional DetNet59, ResNet50, ResNet101, and VGG16 networks and compared them with other high-quality results; our algorithm does a good job in this task. Networks that do not join the dilated bottleneck structure lose some feature information in the deep network, so the detection accuracy is not that good.

The article "Pneumonia Detection Using an Improved Algorithm Based on Faster R-CNN" was published in 2021. Journal: Comput Math Methods Med.

## Figures and Tables

**Figure 1:** Flip processed image.

**Figure 2:** Average gray value distribution histogram.

**Figure 3:** Chest X-ray image preprocessing.

**Figure 4:** The comparison of upsampling and deconvolution.

**Figure 5:** DeepConv-DilatedNet.

**Figure 6:** Network structure for pneumonia detection.

**Figure 7:** Classification loss and regression training loss.

**Figure 8:** The blue and yellow, respectively, represent the AP values before and after filtering the proposals using Soft-NMS, and the numbers on polyline indicates the difference of AP between the two.

**Figure 9:** ROC curve.

**Figure 10:** Precision/recall curve.

**Figure 11:** Comparison of test results of different models.

**Table 1:** Number of marking frames of lesions in the training set and test set.

Dataset/lesion areas in each picture	1	2	3	4
Training set	2068	2628	104	10
Test set	545	629	25	3

**Table 2:** Assessment results for different IoU thresholds.

	AP@0.4	AP@0.5	AP@0.6	AP@0.7	mAP
DetNet59	0.6317	0.4201	0.2068	0.0657	0.3311
ResNet50	0.6066	0.3791	0.1863	0.0513	0.3058
ResNet101	0.5539	0.3508	0.1540	0.0406	0.2748
VGG16	0.5506	0.3559	0.1881	0.0660	0.4210
DeepConv-DilatedNet	**0.6419**	**0.4570**	**0.2732**	**0.0746**	**0.3617**

**Table 3:** Assessment results via Soft-NMS.

Network	mAP@0.4	mAP@0.5	mAP@0.6	mAP@0.7	mAP
DetNet59+Soft-NMS	0.6617	0.4751	0.2638	0.0879	0.3721
DeepConv-DilatedNet+Soft-NMS	**0.6849**	**0.4940**	**0.2863**	**0.1040**	**0.3923**
ResNet50+Soft-NMS	0.6234	0.4268	0.2495	0.0842	0.3460
ResNet101+Soft-NMS	0.5790	0.3992	0.2077	0.0630	0.3122
VGG16+Soft-NMS	0.5925	0.4179	0.2462	0.0940	0.3377

**Table 4:** Comparison of results for different networks.

Network	MS
Mask R-CNN	0.2181
DeepConv-DilatedNet+Soft-NMS	**0.35087**

**Table 5:** Assessment results of chest X-ray.

Network	AP@0.4	AP@0.5	AP@0.6	AP@0.7	mAP
DetNet59+Soft-NMS	0.6343	0.4614	0.2397	0.0875	0.3557
DeepConv-DilatedNet+Soft-NMS	**0.6756**	**0.4796**	**0.2561**	**0.1095**	**0.3802**
ResNet50+Soft-NMS	0.6053	0.4317	0.1884	0.0737	0.3248
ResNet101+Soft-NMS	0.5813	0.4005	0.1656	0.0636	0.3028
VGG16+Soft-NMS	0.5914	0.4109	0.1784	0.0603	0.3103

## Data Availability

The image data used to support the findings of this study can be obtained from the following connection: https://www.kaggle.com/paultimothymooney/chest-xray-pneumonia.
